# Determination of Gypenoside A and Gypenoside XLIX in Rat Plasma by UPLC-MS/MS and Applied to the Pharmacokinetics and Bioavailability

**DOI:** 10.1155/2022/6734408

**Published:** 2022-08-12

**Authors:** Yan He, Qishun Liang, Lvqi Luo, Yifan He, Xueli Huang, Congcong Wen

**Affiliations:** ^1^The Molecular Neuropharmacology Laboratory and the Eye-Brain Research Center, The State Key Laboratory of Ophthalmology, Optometry and Vision Science, Wenzhou Medical University, Wenzhou, China; ^2^Laboratory Animal Center, Wenzhou Medical University, Wenzhou, China; ^3^Analytical and Testing Center, School of Pharmaceutical Sciences, Wenzhou Medical University, Wenzhou, China

## Abstract

In this work, a UPLC-MS/MS method was developed for the determination of gypenoside A and gypenoside XLIX in rat plasma. For chromatographic separation, a UPLC BEH C18 column was employed, the mobile phase comprised acetonitrile: water (w/0.1% formic acid), and the elution time was 4 min. Detection of each compound was enabled by electrospray ionization in negative-ion mode, and quantitative analysis was enabled by operating in multiple reaction monitoring (MRM) mode by monitoring the transitions of m/z 897.5⟶403.3 for gypenoside A, m/z 1045.5⟶118.9 for gypenoside XLIX, and m/z 825.4⟶617.5 for the internal standard. The calibration curves for gypenoside A and gypenoside XLIX demonstrated excellent linearity (*r* > 0.995) over the range of 2–3000 ng/mL. The intraday and interday precisions of gypenoside A and gypenoside XLIX were within 14.9%, the intraday and interday accuracies ranged from 90.1% to 113.9%, the recoveries were all greater than 88.3%, and the matrix effect ranged from 87.1% to 94.1%. The developed method was successfully applied in the determination of the pharmacokinetics of gypenoside A and gypenoside XLIX. Gypenoside A and gypenoside XLIX had very short half-lives in rats, with oral *t*_1/2z_ of 1.4 ± 0.2 h and 1.8 ± 0.6 h, respectively, and low bioavailabilities (0.90% and 0.14%, respectively).

## 1. Introduction

*Gynostemma pentaphyllum* Makino, also known as five-leaf ginseng and horse chestnut gall [1], is a perennial trailing herb and member of the Cucurbitaceae family of flowering plants [2, 3]. *Gynostemma pentaphyllum* Makino is known to produce a variety of dammarane-type gypenosides [4–6], which have been shown to display antioxidant, antiinflammatory, immunogenic, hypolipidemic, and hypoglycemic effects [7–11]. Gypenosides have also demonstrated protective effects against neurological diseases, such as Alzheimer's disease, Parkinson's disease, depression, and hypoxic brain injury [12–14].

Gypenoside A and gypenoside XLIX are the two main saponins found in *Gynostemma pentaphyllum* [15, 16] and have been isolated from the plant and purified by LC-MS/MS. Guo et al. performed a solid-phase extraction method and developed an LC-MS/MS method to detect gypenoside XLIX in rat plasma [15]. They then studied the rat pharmacokinetics of gypenoside XLIX after intravenous administration. Hu et al. developed a quantitative UPLC-MS method to detect gypenoside A in rat plasma [17]. Each sample required 5 min, the proteins were precipitated with methanol to avoid interference from matrix effects, and the gypenoside A concentration in rats was determined after oral administration of Gelanxinning soft capsules. However, both methods only analyzed the *in vivo* concentration of gypenoside A or gypenoside XLIX separately, and neither detected them simultaneously nor did they conduct bioavailability studies.

In this paper, we developed a UPLC-MS/MS method to enable the simultaneous determination of gypenoside A and gypenoside XLIX in rat plasma and then utilized the method to study the pharmacokinetics of both gypenosides under different administration routes (oral and intravenous administration) to determine their bioavailability.

## 2. Experimental

### 2.1. Reagents

Gypenoside A (purity ≥98%, Figure 1(a)), gypenoside XLIX (purity ≥98%, Figure 1(b)), and saikosaponin B2 (internal standard, purity ≥98%, Figure 1(c)) were purchased from Chengdu Mansite Pharmaceutical Co., Ltd. (Chengdu, China). HPLC-grade methanol and acetonitrile were purchased from Merck KGaA (Darmstadt, Germany). Ultrapure water (resistance >18 mΩ) was used to prepare all solutions in this study and was prepared using a Milli-Q purification system (Bedford, MA, USA).

### 2.2. Instrument Conditions

An ACQUITY I-Class ultraperformance liquid chromatography system coupled with a Waters XEVO TQ-S microtriple quadrupole tandem mass spectrometer was employed for the detection of gypenosides A and XLIX. The ACQUITY I-Class UPLC system was equipped with a UPLC BEH C18 column (50 mm × 2.1 mm, 1.7 *μ*m), and the column temperature was set to 40°C. The mobile phase consisted of a gradient elution of acetonitrile: water (w/0.1% formic acid), the flow rate was 0.4 mL/min, and the elution time was 4 min. Gradient elution profile consisted of 10% acetonitrile, 0–0.2 min; 10–70% acetonitrile, 0.2–1.0 min; 70–90% acetonitrile, 1.0–2.5 min; 90–10% acetonitrile, 2.5–2.8 min; 10% acetonitrile, 2.8–4.0 min.

For the mass spectrometer, nitrogen was used as the cone gas (50 L/h flow rate) and desolvation gas (1000 L/h flow rate). The capillary voltage was set to 3.2 kV, the ion source temperature was 145°C, and the desolvation temperature was 500°C. The mass spectrometer was operated in electrospray (ESI) negative-ion mode, and the quantitation of the two gypenosides was enabled by operating in multiple reaction monitoring modes (MRM) by monitoring the transitions of m/z 897.5⟶403.3 (cone voltage 76 V, collision voltage 40 V) for gypenoside A (Figure 2(a)), m/z 1045.5⟶118.9 (cone voltage 70 V, collision voltage 70 V) for gypenoside XLIX (Figure 2(b)), and m/z 825.4⟶617.5 (cone voltage 22 V, collision voltage 42 V) for the internal standard.

### 2.3. Standard Curve

Stock solutions (500 *µ*g/mL) of gypenoside A, gypenoside XLIX, and the internal standard were prepared in methanol. The stock solutions were diluted with methanol to obtain working solutions of gypenoside A and gypenoside XLIX at a range of concentrations (20, 100, 200, 500, 2000, 5000, 10000, 20000, and 30000 ng/mL). All stock and working solutions were stored at 4°C. The gypenoside A and gypenoside XLIX working solutions were diluted into blank rat plasma to obtain a series of solutions of the two gypenosides in rat plasma with concentrations of 2, 10, 20, 50, 200, 500, 1000, 2000, and 3000 ng/mL. Quality control (QC) samples were also prepared in blank rat plasma at different concentrations (5, 250, and 2500 ng/mL) under the same conditions.

### 2.4. Sample Preparation

To prepare the plasma samples, 50 *μ*L of rat plasma was added to a 1.5 mL Eppendorf tube, to which 150 *μ*L of acetonitrile-methanol (9 : 1, v/v) (containing 100 ng/mL of the internal standard) was added. The solutions were vortexed for 1.0 min and centrifuged at 13000 rpm for 10 min at 4°C. An aliquot (100 *μ*L) of the supernatant was transferred to a lined tube of the injection bottle, and 3 *μ*L of the solution was injected into the UPLC for UPLC-MS/MS analysis.

### 2.5. Pharmacokinetics

Sprague Dawley (SD) rats (male, 220–250 g) were obtained from the Animal Experiment Center of Wenzhou Medical University (Wenzhou, China). All experimental procedures and protocols were approved by the Animal Care Committee of Wenzhou Medical University. Six rats were administered gypenoside A was administered intravenously (iv, 1 mg/kg) and orally (po, 5 mg/kg), and another six rats were administered the same dosages of gypenoside XLIX, for a total of 12 rats. At 0.0833, 0.25, 1, 2, 4, 6 h (for gypenoside A) and 0.0833, 0.25, 1, 2, 4, 6, 8, 12 h (for gypenoside XLIX) postadministration, 0.2 mL of blood was collected from the caudal (tail) vein into heparinized Eppendorf tubes, which were centrifuged at 13000 rpm for 10 min. Then, 50 *μ*L of the plasma (top-most layer) was transferred to a 1.5 mL Eppendorf tube and stored at –80°C until analysis of the pharmacokinetic parameters, which were statistically calculated using the pharmacokinetic DAS 2.0 software. The formula for absolute bioavailability was AUC for oral administration/AUC for intravenous administration × 100%.

## 3. Results and Discussion

### 3.1. Method Development

The mass spectrometry conditions were obtained after optimizing the spray needle voltage, drying gas temperature, capillary voltage, and collision energy [18–21]. Comparing the positive and negative modes, gypenoside A and gypenoside XLIX were best suited for detection in ESI negative-ion mode because the sensitivity was significantly higher than detection in other modes. Gypenoside A and gypenoside XLIX were prepared in rat blank plasma at a concentration of 100 ng/mL. During the method development, a variety of different solvents and solvent mixtures were assessed for their ability to efficiently precipitate the proteins in the rat plasma. Acetonitrile, methanol-acetonitrile (1 : 9, v/v), 10% trichloroacetic acid, methanol-acetonitrile (1 : 1, v/v), and methanol were employed, and it was determined that methanol-acetonitrile (1 : 9, v/v) had the highest extraction efficiency, so it was chosen as the solvent for the protein precipitation step.

### 3.2. Selectivity

As shown in Figure 3, the retention times of gypenoside A, gypenoside XLIX, and the internal standard were 1.86, 1.72, and 1.91 min, respectively, and there was no interference from the endogenous components within the plasma, indicating that the developed method was highly selective for the two natural compounds.

### 3.3. Standard Curve

The calibration curves of gypenoside A and gypenoside XLIX in rat plasma that were generated over the concentration range of 2–3000 ng/mL demonstrated excellent linearity, indicating that they could reliably be used for calculating the concentration of the natural compounds in the rat plasma. The regression equation for gypenoside A was *y*1 = 0.0096*x*1 + 0.0023 (*R*^2^ = 0.9984), wherein x1 represented the concentration of gypenoside A in the plasma, and y1 represented the ratio of the peak area of gypenoside A to the internal standard. The regression equation for gypenoside XLIX was *y*2 = 0.0024*x*2 + 0.0014 (*R*^2^ = 0.9971), wherein x2 represented the concentration of gypenoside XLIX in plasma, and y2 represented the ratio of the peak area of gypenoside XLIX to the internal standard. Based on these two equations, the lower limit of quantification of gypenoside A and gypenoside XLIX in rat plasma was 2 ng/mL, and the detection limit was 1 ng/mL.

### 3.4. Precision, Accuracy, Recovery, and Matrix Effects

The intraday and interday precisions of gypenoside A were within 14.9%, the intraday and interday accuracies were 90.1–107.5%, the recovery was greater than 88.3%, and the matrix effects were 87.1–93.9%. The intra- and interday precisions of gypenoside XLIX were within 12.9%, the intra- and interday accuracies were 91.8–113.9%, the recovery was greater than 93.2%, and the matrix effects were in the range of 89.3–94.1% (Table 1).

### 3.5. Stability

The accuracy of gypenoside A was between 92.2% and 110.3%, and the RSD was within 14.8%; the accuracy of gypenoside XLIX was between 87.9% and 112.2%, and the RSD was within 14.5% (Table 2). These results indicated that gypenoside A and gypenoside XLIX had excellent stability.

### 3.6. Pharmacokinetic Studies

The noncompartmental model was used to fit the main pharmacokinetic parameters (Table 3), and the concentration-time curves for gypenoside A and gypenoside XLIX in rat plasma are shown in Figure 4. After intravenous administration, the half-lives (*t*_1/2z_) of gypenoside A and gypenoside XLIX in the rats were 0.8 ± 0.2 h and 1.6 ± 1.7 h, respectively, while the oral *t*_1/2z_ were 1.4 ± 0.2 h and 1.8 ± 0.6 h, respectively, indicating that the compounds were metabolized very quickly. The *t*_1/2_ of gypenoside A in rats reported in the literature was 6.247 ± 2.039 h [17], which is significantly longer than the values we reported, but this difference was likely due to the different dosage forms. However, the *t*_1/2_ of gypenoside XLIX in rats reported in the literature (3.17 ± 1.01) *h* was closer to the values we calculated [15]. Based on the pharmacokinetics data, gypenoside A and gypenoside XLIX had very low oral bioavailabilities of 0.90% and 0.14%, respectively, indicating that the concentration of the drug in systemic circulation was low.

## 4. Conclusion

In this study, a UPLC-MS/MS method was established for the determination of gypenoside A and gypenoside XLIX in rat plasma. The UPLC-MS/MS method required only 4 min for each sample, and a simple and inexpensive protein precipitation method was used. The accuracy, precision, selectivity, and linearity of this method were highly robust, corroborating the application of this method in studying the pharmacokinetics and bioavailability of these compounds and others alike in rats.

## Figures and Tables

**Figure 1:** Chemical structure of gypenoside A (a), gypenoside XLIX (b), and saikosaponin B2 (c), the internal standard.

**Figure 2:** Mass spectra of gypenoside A (a) and gypenoside XLIX (b).

**Figure 3:** UPLC-MS/MS chromatograms of gypenoside A, gypenoside XLIX, and the internal standard in rat plasma (a) and blank rat plasma spiked with gypenoside A, gypenoside XLIX, and internal standard (b).

**Figure 4:** The concentration-time curve of rats after intravenous (iv, 1 mg/kg) and oral (po, 5 mg/kg) administration of gypenoside A (a) and gypenoside XLIX (b).

**Table 1:** Accuracy, precision, matrix effect, and recovery of gypenoside A and gypenoside XLIX in rat plasma.

Compound	Concentration (ng/mL)	Accuracy (%)		Precision (RSD%)		Matrix effect (%)	Recovery (%)
		Intraday	Interday	Intraday	Interday		
Gypenoside A	2	90.1	107.5	13.8	14.9	89.9	92.7
	5	103.2	90.5	7.0	6.4	93.5	88.3
	250	100.0	102.9	8.5	7.9	93.9	95.0
	2500	101.8	103.3	6.1	9.9	87.1	89.4
	2	91.8	113.9	10.4	12.9	90.4	97.1

Gypenoside XLIX	5	108.9	94.2	8.1	10.4	92.9	94.4
	250	106.2	106.1	8.1	11.3	94.1	93.2
	2500	99.3	94.2	6.1	4.4	89.3	98.2

**Table 2:** Stability of gypenoside A and gypenoside XLIX in rat plasma (%).

Compound	Concentration (ng/mL)	Autosampler (4°C, 12 h)		Ambient (2 h)		−20°C (30 d)		Freeze-thaw	
		Accuracy	RSD	Accuracy	RSD	Accuracy	RSD	Accuracy	RSD
Gypenoside A	5	101.9	7.8	93.7	9.2	102.7	13.3	110.3	14.8
	250	100.5	2.8	99.9	5.3	93.8	7.2	108.6	7.2
	2500	96.6	5.6	106.0	5.6	99.8	5.9	92.2	6.0
	5	101.1	11.7	107.7	11.5	112.2	14.5	91.2	13.3

Gypenoside XLIX	250	108.6	8.4	97.4	6.5	90.7	7.9	87.9	13.0
	2500	99.5	8.0	95.5	8.8	88.0	1.4	103.9	9.5

**Table 3:** Main pharmacokinetic parameters after intravenous (iv) and oral (po) administration of gypenoside A and gypenoside XLIX in rats.

Compound	Group	AUC_(0-*t*)_ (ng/mL·h)	AUC_(0-∞)_ (ng/mL·h)	*t*_1/2z_ (h)	CL_z/F_ (L/h/kg)	*V*_z/F_ (L/kg)	*C*_max_ (ng/mL)
Gypenoside A	Po, 5 mg/kg	14.9 ± 2.4	15.9 ± 2.5	1.4 ± 0.2	319.9 ± 49.8	665.4 ± 161.4	8.6 ± 1.3
	Iv, 1 mg/kg	332.9 ± 31.2	334.3 ± 32.2	0.8 ± 0.2	3.0 ± 0.3	3.3 ± 0.7	621.9 ± 36.2

Gypenoside XLIX	Po, 5 mg/kg	13.7 ± 2.5	15.4 ± 2.2	1.8 ± 0.6	330.8 ± 52.7	879.8 ± 345.0	8.1 ± 0.9
	Iv, 1 mg/kg	1923.5 ± 62.5	1926.6 ± 62.3	1.6 ± 1.7	0.52 ± 0.02	1.2 ± 1.3	2201.9 ± 211.6

## Data Availability

The data used to support the findings of this study are included within the article.
